This article has been retracted.

# Hotspot Mining in the Field of Library and Information Science under the Environment of Big Data

**DOI:** 10.1155/2022/2802835

**Published:** 2022-07-31

**Authors:** Shujie Jiang

**Affiliations:** Nanyang Normal University, Nanyang 473061, China

## Abstract

Currently, with the implementation of big data strategies in countries all over the world, big data has achieved vigorous development in various fields. Big data research and application practices have also rapidly attracted the attention of the library and information field. *Objective*. The study explored the current state of research and research hotspots of big data in the library and information field and further discussed the future research trends. *Methods*. In the CNKI database, 16 CSSCI source journals in the discipline of library information and digital library were selected as data sources, and the relevant literature was retrieved with the theme of “big data.” The collected literature was excluded and expanded according to the citation relationship. Then, with the help of Bicomb and SPSS, co-word analysis and cluster analysis would be carried out on these literature results. *Results*. According to the findings of the data analysis, the research hotspots on the topic mainly focus on five major research themes, namely, big data and smart library, big data and intelligence research, data mining and cloud computing, big data and information analysis, and library innovation and services. *Limitations*. At present, the research scope and coverage on this topic are wide, which leads to the research still staying at the macro level. *Conclusions*. Big data research will remain one of the hotspots in the future. However, the most study is still limited to the perspective of library and information and has not yet analyzed the research status, research hotspots, and development trends in this field from the perspective of big data knowledge structure. Moreover, machine learning, artificial intelligence, knowledge services, AR, and VR may be new directions for future attention and development.

## 1. Introduction

The emergence of intelligent technology tools has ushered in the fourth paradigm of scientific research, which is characterized by data-intensive research [1]. In this context, big data provides rich “nutrients” for research in various disciplines [2–4]. Data-driven approaches and concepts have become the new engine of big data utilization, gradually penetrating scientific research in various disciplines [5]. The concept of big data was first formally introduced by “Nature” in 2008. Once it was introduced, it became a research hotspot in various fields at a fast speed. Scholars have started to explore the application value of big data in various fields from different perspectives [6, 7]. Of course, the field of library and information dealing with data, information, and documents is no exception. Driven by big data, scholars in this field have also rapidly joined the ranks of big data research. Big data research has reshaped people's understanding of data, and also promoted the transformation of academic research from traditional theoretical empirical and computational research models to data-driven research paradigms [8]. Therefore, the arrival of the big data era seems to have had a considerable effect on the evolution of the library and information domain. As pioneers in the implementation of developing information science and computational technology, some scholars of library and information have also promptly changed their concepts, reshaped big data thinking, and fully integrated big data technology with research in their field to carry out relevant thematic research work [9]. It can be said that, driven by big data, the work mode and the work content of the library and information field have ushered in unprecedented new challenges, and the traditional work mode of mainly collecting and analyzing information can hardly match the development demands of the growing era. The focus of the work in the library and information domain began to change from literature and information to data.

The library and information science have been associated with data, information, and intelligence from the very beginning of their development. Its essence is to achieve order by reorganizing and processing various types of data and knowledge. Therefore, whether it is the research of library and information or big data research, it is strongly intertwined with data support. This has attracted many scholars to start exploring the impact of big data on the development of library and information. Representative studies include examining the effect of big data on intelligence research from the research process [10], and putting forward the framework of intelligence system under the big data paradigm [11], intelligence theory [12], intelligence methods and technology system [13], intelligence discipline positioning [14], and the change or construction of intelligence principles, methods and practices [15], respectively. With the increasing number of related research results, summarizing and analyzing the hot issues in the research field has also become an urgent task. And some scholars have already attempted the related research work and achieved certain results. Literature [16, 17] aimed at the research results on big data in the library and information science, and used relevant bibliometric analysis software to visually analyze the research topics of this discipline. In this way, the hotspots in the research topics are excavated and the potential development trends are summarized. In summary, the research hotspots in the current field are mainly focused on several aspects such as intelligent library [18], data mining [19], intelligence research [20], and knowledge services.

From the current research, many researchers have presented reasonably extensive research on the above topic, and have achieved richer research results. It has built a good basis for mastering the overall research direction of the domestic library and information field, but it still needs to be further expanded. First, the existing research does not analyze the research status, research hotspots, and development trend of the field from the perspective of the overall knowledge structure of big data research. Second, the acquisition of research samples and the determination of high-frequency keywords are still based on subjective experience, lacking a scientific basis. This is easy to have some influence on the analysis results, and cannot fully reveal the current situation of big data research in the library and information field. Therefore, in order to more accurately grasp the current situation and hotspots on our research topics, the innovative work of this research is as follows: firstly, the literature in the related field included in the CNKI database was searched with the theme of “big data,” and the collected literature was used as a sample source for preliminary collation and analysis. Secondly, Bicomb and SPSS were utilized to analyze the results of the processed literature for co-word analysis and cluster analysis. Finally, by clustering high-impact literature to identify research frontier topics, the research hotspots of library and information disciplines are driven by big data are revealed. Besides, we draw relevant conclusions to provide help and reference for research in this field.

## 2. Research Methodology

### 2.1. Data Sources

CSSCI source journals are one of the most academically influential representative journals in the field of humanities and social sciences in China. The studies published in them have high academic value and scientific research level, which can fully reflect the research level and strength of a discipline. Therefore, this study selected 16 CSSCI journals in the related field (see Table 1 for details). Then a subject search was conducted in the CNKI database to obtain the data sources. The detailed search process is as follows: retrieval subject = “big data, retrieval subject = “library information and digital library,” literature sources are set to 16 journals in Table 1, time span: 2011–2020.1536 results were retrieved. After analyzing and sorting the search results and eliminating the irrelevant papers, a total of 1420 research papers were obtained.

As can be seen from Table 1, during the period of 2011–2020, several journals of “Library and Information Service”, “Information studies: Theory and Application”, “Researches In Library Science”, “Information Science”, “Journal of Modern Information”, “Library and Information” have the largest number of studies published on the research topic, with a total number of 1001, accounting for 65.17% of all research results. In addition, more than 200 studies on big data research have been published in the two journals “Library and Information Service” and “Information studies: Theory and Application.” On the contrary, the number of studies issued in the journals of “Library Development”, “Journal of Academic Libraries”, “Library Tribune”, “Journal of the National Library of China” and “Journal of Library Science in China” are less than 50, and the least number is only 21. In general, the quantity of scientific publications in library science journals is far behind that of intelligence journals on the research topic. This also reflects the fact that big data research is more popular and more emphasized in intelligence journals than in library journals.

### 2.2. Methodology

In this study, we will mainly use Bicomb and SPSS to analyze the data of the collected effective literature. First, the keywords in the literature are cleaned and standardized by Bicomb software in order to identify the high-frequency keywords in our research topic. And based on this, the co-occurrence matrix of high-frequency keywords will be constructed. Second, the obtained co-occurrence matrix will be converted into a dissimilarity matrix of high-frequency keywords by using SPSS software, and then cluster analyses are conducted to obtain a dendrogram of cluster results. The co-occurrence matrix of high-frequency keywords can help us to clearly understand the correlation among the various research topics. Then the cluster analysis method is utilized to further classify these high-frequency keywords, and the multiple topics with strong correlations are grouped into a relatively independent cluster. The two research methods used in our research are described below, respectively.

As a content analysis method, the co-word analysis determines the relevance between a pair of keywords that can indicate the topic by counting how many times they occur together in the literature [21]. In other words, the relevance between any two subject terms or keywords is positively correlated with the number of times they co-occur in a piece of literature. That is, the higher the number of co-occurrences, the closer the relationship between them. On the contrary, if the number of co-occurrences is zero, it indicates that there is no relationship between these two words. Zipf's law clearly states that the co-occurrence matrix will have a demarcation point between high-frequency words and low-frequency words, which is called the high-frequency word threshold. Its calculation method is shown in

(1) $$\begin{array}{c} K=\frac{-1+\sqrt{1+8N_{1}}}{2}. \end{array}$$

Here, *N*_1_ denotes the total number of keywords that have appeared only once. In order to better analyze the themes of the research area, the keyword co-occurrence matrix was constructed by using co-word analysis method. By screening the number of high-frequency words, the corresponding *K* × *K* matrix was constructed, and the matrix calculation was performed to calculate the number of co-occurrence between each high-frequency word of the matrix. The detailed calculation process is shown in

(2) $$\begin{array}{c} y=\left\{\begin{array}{cc} +1, & \text{there is co}-\text{occurrence of a and b keywords,}\\ 0, & \text{there is no co}-\text{occurrence of a and b keywords.} \end{array}\right. \end{array}$$

Suppose there are four high-frequency words: A, B, C, and D. Then a 4 × 4 co-occurrence matrix needs to be constructed, as in

(3) $$\begin{array}{c} \begin{array}{ccccc} - & A & B & C & D\\ A & 0 & 1 & 2 & 1\\ B & 1 & 0 & 1 & 1\\ C & 2 & 1 & 0 & 1\\ D & 1 & 1 & 1 & 0 \end{array}. \end{array}$$

In formula (3), each value means the number of times any two keywords occur together in the same literature. The larger the value, the more times the two words appear together, and the stronger the correlation between them. For instance, keyword A and keyword C occur together twice; and A and B, A and D co-occur once, respectively. This shows that the correlation between A and C is stronger compared to A and B or A and D. In addition, formula (3) was further transformed for the purpose of later data statistics and analysis, as illustrated in Table 2.

Then, the Ochiai coefficient method was utilized to calculate the keyword similarity matrix, and the conversion process is shown in

(4) $$\begin{array}{c} O_{ab}=\frac{N_{ab}}{\sqrt{N_{a}}\times \sqrt{N_{b}}}. \end{array}$$

Here, *O*_*ab*_ represents the co-occurrence similarity between keyword *a* and keyword *b*. *N*_*ab*_ indicates the total number of co-occurrence of *a* and *b*, *N*_*a*_ stands for the number of occurrences of *a* alone, and *N*_*b*_ indicates the number of occurrences of *b* alone.

In addition, as a classification method, the cluster analysis method has unique advantages in mining the hot topics in different areas. Based on the keyword co-occurrence matrix, cluster analysis uses the degree of association between a pair of keywords to classify them [22], which in turn reveals the research hotspots and changing trends of the topic. In the clustering process, the classification is based on the distance between the two keywords. Multiple keywords that are closer and more related are clustered into a relatively independent cluster.

## 3. Data Analysis

### 3.1. Analysis of the Number of Papers Issued

To a certain extent, the distribution trend of annual publication volume may be able to give an expression of the changing trend of research hotspots in a particular field at different periods. In view of this, the study organizes and analyzes the effective literature data retrieved. The number of publications in different years is presented in a line graph, and the distribution trend of the publication volume with the theme of “big data” in the research field from 2011 to 2020 is obtained, as illustrated in Figure 1.

From Figure 1, we can find that the number of the studies issued on the research topic has shown a steady growth trend from 2011 to 2020. The development process may be roughly separated into two phases. The first phase is the preliminary exploration period before 2014. During this period, the number of annual publications was below 50, and only 1 in 2011, which was relatively small. As the research on big data in China just started in this period, it has not yet attracted enough attention from scholars in the related field. However, the second phase (from 2014 to the present) is the hot time period. The number of studies published in this period has been growing rapidly. In particular, the peak period is reached in 2019, with 271 papers published. Then the number of research results decreases in 2020, entering a period of relative saturation.

### 3.2. High Frequency Keyword Analysis

Keywords are a high summary of the research content of a paper and can fully reflect the research topic characteristics of the paper. The word frequency statistics and co-word analysis of keywords are helpful to mine the research topics in our research field. First, the sample data collected from CNKI were imported into Bicomb software to obtain the keywords appearing in the papers. Then, data filtering and synonym merging are further performed on the extracted keywords to extract effective topic keywords. Finally, using the Bicomb software, the top 30 high-frequency keywords with frequency ≧5 were selected as the main research objects. The statistical results are illustrated in Table 3.

Analyzing the data in Table 3, we can find that “big data” and “library” are the two keywords with the highest frequency in academic research, and they are the hot spots in the research field. This also means that the research mainly revolves around “big data” and gradually extends to related fields, resulting in a series of other keywords, such as “intelligent library,” “digital library,” “cloud library.” Second, high-frequency keywords such as “cloud computing,” “data mining,” “data analysis,” “data processing,” “Internet of Things,” and “unstructured data” represent new technical means. It reflects that while scholars in the research field are conducting theoretical innovation research, they also integrate a variety of advanced technologies, especially emerging technologies, to promote the reform and development of the library and information. In addition, keywords such as “knowledge service,” “personalized service,” “knowledge consultation,” “information resources,” “information analysis” and “information technology” appear frequently. It reflects that in the big data environment, research on data storage, data analysis, data processing, and information services has attracted great attention from scholars.

Based on Table 3, the research will also use Bicomb software to construct a co-occurrence matrix of the top 30 high-frequency keywords with a size of 30 × 30, as shown in Table 4. However, considering that the number of co-occurrences of each keyword pair may differ greatly and cannot reflect the direct connection between the keywords, the similarity matrix of high-frequency keywords is further constructed. In this study, the Ochiia coefficients are calculated according to formula (4), and the co-occurrence matrix is converted into the corresponding similarity matrix, as shown in Table 5. The values in the similarity matrix are in the interval of [0, 1]. Similar to the co-occurrence matrix principle, the closer the value in the similarity matrix is to 1, the higher the similarity between two keywords. On the contrary, the similarity between them is lower. In addition, because there are too many 0 values in the similarity matrix, errors are prone to occur in the statistical results. Therefore, to ensure the effectiveness of cluster analysis, the similarity matrix of hot keywords is converted into a dissimilarity matrix, as illustrated in Table 6. In contrast to the similarity matrix, the larger the value in the dissimilarity matrix, the lower the similarity between the two keywords. Due to the limitation of space, Tables 4–6 present only partial statistical results.

Analyzing the data in the above three tables, we may find that among the top 30 high-frequency key species, “big data” and “smart library,” “big data” and “data mining,” “big data” and “cloud computing,” “and library” and “big data era” appear together most frequently with more than 10 times. And the value of the above pairs of keywords in the similarity matrix is closer to 1. This indicates that there is a stronger correlation between these keywords.

### 3.3. Cluster Analysis

Clustering analysis can classify each pair of keywords into different clusters according to their distances from each other. The closer the distance, the more related the keywords will be grouped into the same cluster. And there will be large differences between different clusters. Therefore, in order to dig out the research hotspots of our research topic, the dissimilarity matrix of high-frequency keywords is imported into SPSS for clustering analysis. In SPSS, select “Systematic Clustering Analysis,” and then set the clustering method to “Intergroup Connection” to generate a clustering analysis tree diagram of hotspot keywords on the topic of big data in the field, as illustrated in Figure 2.

As shown in Figure 2, the hot keywords on the research topic are mainly focused on the following five categories: the first category focuses on library research, such as digital library, intelligent library, cloud library. The second category is mainly related to intelligence research, including intelligence, competitive intelligence, bibliometrics. The third category is mostly about big data, cloud computing, the Internet of Things, data mining, unstructured data, and so on. The fourth category is big data and information analysis, and information processing. The fifth category is mainly related to innovative library services driven by big data, such as library services, knowledge services, personalized services, information services.

## 4. Hotspot Exploration

On the basis of the research analysis, this study will summarize and classify the hotspots in the research field from the following five aspects, so as to supply a certain reference for further research in related fields.

### 4.1. Big Data and Smart Library

In the era of big data, the smart library will become a new mode of library development in the future. It can be said that a smart library is at a higher stage than a digital library, mobile library, or cloud library. It relies on intelligent technologies and systems and uses massive data resources as “nutrients” to realize the interconnection between readers, books (or documents), and libraries, so as to provide personalized services for readers and greatly improve their service experience. The research in the related field has also made some progress on this topic. For example, the literature [23] designed a development plan for a smart library system platform with the help of cloud computing and big data technologies. The platform incorporates data collection and management, real-time state of affairs awareness, and intelligent services in one. At present, China has not built a smart library in the real sense. However, Wuhan University, Nanjing University, and other universities have started to make preliminary exploration into the construction of smart libraries. It is believed that more and more academic institutes will participate in the research and development team of smart libraries in the future under the influence of the practice of the libraries of universities. Therefore, smart libraries are bound to be one of the hotspots in the research field.

### 4.2. Big Data and Intelligence Research

Data is almost inextricably linked to intelligence research. Therefore, in the context of big data, librarians and information scientists place an emphasis on integrating intelligence research with technological tools like big data, data mining, and the IoT in order to create a new scientific and technological intelligence system. For example, literature [24] proposes a framework for intelligence analysis on the basis of the framework structure of big data, aiming to provide users with a basis for decision making. The framework also has functions such as analysis of public opinion hotspots. Competitive intelligence is also one of the important contents of intelligence research. In the current context, competitive intelligence is closely related to national development and national security and has always occupied an important position among the research topics in the research field.

### 4.3. Cloud Computing and Data Mining

It has been proved that technologies related to big data have made vigorous development in the library and information area, including cloud computing, data mining, IoT, and so on. With the maturation of cloud computing theory and technology in the latest years, its application scope in the research field has grown significantly, covering data storage, data computing, resource sharing, data management, and so on. It can be said that the research on cloud computing and big data are complementary to each other. Cloud computing application research based on big data has received much interest and has been widely used in the integration of digital library resources. In addition, big data mining technology has also achieved fruitful research results in our research field, and it has played an important value in library resource construction, library personalized services, etc.

### 4.4. Big Data and Information Analysis

Information analysis refers to the information labor process of in-depth thinking processing and analysis of a large amount of relevant information according to the needs of specific problems and forming new information that is helpful for problem-solving. Data is expanding at a breakneck pace in the current environment. Therefore, in the face of these diverse and large-scale unstructured data, the traditional sample information analysis methods have been difficult to uncover the latent values in big data. Therefore, a new way of processing and analyzing these huge data sets is required, so as to uncover the latent relationships in the data. Therefore, big data will be not only a data revolution but also a thinking change. The concept of big data has had a significant influence on information processing methods in the field to some extent and promoted its transformation from the traditional information analysis method to a more accurate and efficient direction.

### 4.5. Library Innovation and Services

In the current environment, libraries have both opportunities and challenges. Many scholars have proposed that libraries should attach importance to user data, mine massive data, deepen service innovation, and provide readers with personalized services. In the era of information explosion, effective information is easily annihilated by a variety of massive information, and the cost for users to obtain effective information is greatly increased. In this context, knowledge service has become one of the key businesses of the library, so it has also become a research hotspot in the research field. Knowledge service is developed on the basis of document service and information service. Traditional document services and information services only provide readers or users with information retrieval, document retrieval, and other services. The knowledge service based on big data is different. The service resources and service scale it provides are larger, and it can provide customized and personalized services for users according to their needs. Therefore, the knowledge products provided by them often have a higher intellectual level, thus meeting the more complex knowledge needs of readers.

## 5. Conclusion

Driven by big data, the research work in the library and information field in our country is in the process of continuous change and innovation. Scholars have been able to change their thinking in time, closely integrate with big data technology, and seek innovation and breakthroughs in theory and practice. As a result, fruitful research results have emerged. In this study, using CNKI as the data source, we conduct an in-depth analysis of 1460 relevant literature published in 16 representative journals of CSSCI from 2011 to 2020. On this basis, using co-word analysis and cluster analysis, the research status, research hotspots, and trend changes in the library and information field under the impact of big data are analyzed from multiple perspectives. Finally, the following insights are drawn: First, the hotspots in the research field mainly focus on five themes, which are big data and smart library, big data and intelligence research, data mining and cloud computing, big data and information analysis, and library innovation and services. Second, as a result of the influence of intelligent systems, the research hotspots in the domestic library and information field in recent years have gradually shifted from digital libraries, intelligence analyses, and information services to knowledge services and intelligent libraries, which is likely to become a new knowledge growth point in the research field. Third, Scholars' research on our topic is no longer purely theoretical, but they also place a high value on research into big data-related technologies and applications. Although the research presented in our work has some practical implications and can provide useful references for promoting high-quality academic development in the domestic library and information field driven by big data. It is not without limitations. Because of the huge amount of literature referring to big data research, the current research topics and development trends in the library and information field can only be analyzed from a macro perspective. In addition, the selection of hot keywords does not have a more adequate theoretical basis and is somewhat subjective. Therefore, future methods to effectively classify high-frequency words need to be further studied.

## Figures and Tables

**Figure 1:** The distribution trend of the publication volume with the theme of “big data” in the library and information science in China from 2011 to 2020.

**Figure 2:** The clustering analysis tree diagram of hotspot keywords on the research topic.

**Table 1:** Distribution of retrieved studies among 16 journals.

Number	Journals	Number of studies issued	Percentage
1	*Library and Information Service*	217	14.13
2	*Information studies: Theory and Application*	203	13.22
3	*Researches in Library Science*	162	10.55
4	*Information Science*	151	9.83
5	*Journal of Modern Information*	149	9.70
6	*Library and Information*	119	7.75
7	*Journal of Intelligence*	97	6.32
8	*Information and Documentation Services*	88	5.73
9	*Library Journal*	78	5.08
10	*Journal of the China Society for Scientific and Technical Information*	59	3.84
11	*Document, Information and Knowledge*	57	3.52
12	*Library Development*	47	3.06
13	*Journal of Academic Libraries*	34	2.21
14	*Library Tribune*	33	2.15
15	*Journal of the National Library of China*	24	1.56
16	*Journal of Library Science in China*	21	1.37

**Table 2:** The weight results of formula (3).

Source	Target	Weight
A	B	1
A	C	2
A	D	1
B	C	1
B	D	1
C	D	1

**Table 3:** The top 30 high-frequency keywords.

Keywords	Frequency
Big data	241
Library	135
Smart library	63
Big data era	55
Data mining	43
Information service	32
Cloud computing	30
Digital library	28
Knowledge service	25
Data analysis	22
Data processing	18
Competitive intelligence	18
Library service	15
Cloud library	12
Personalized service	11
Digital resources	10
Public library	10
Knowledge consultation	9
Internet of things	8
Intelligence analysis	8
Unstructured data	7
Resource construction	7
Information resource	6
Information analysis	6
Information technology	6
Bibliometrics	5
Library big data	5
Data environment	5
Information science	5
Big data knowledge service	5

**Table 4:** Co-occurrence matrix of the top 30 high-frequency keywords (partial).

	Big data	Library	Smart library	Big data era	Data mining	Information service	Cloud computing	Digital library
Big data	241	0	10	5	12	9	12	8
Library	0	135	9	12	1	4	0	6
Smart library	10	9	63	7	6	5	6	0
Big data era	5	12	7	55	8	3	2	1
Data mining	12	1	6	8	43	4	2	0
Information service	9	4	5	3	4	32	0	3
Cloud computing	12	0	6	2	2	0	30	1
Digital library	8	6	0	1	0	3	1	28

**Table 5:** Similarity matrix of the top 30 high-frequency keywords (partial).

	Big data	Library	Smart library	Big data era	Data mining	Information service	Cloud computing	Digital library
Big data	1.0000	0.0000	0.0812	0.0434	0.1179	0.1025	0.1411	0.0972
Library		1.0000	0.0976	0.1393	0.0131	0.0609	0.0000	0.0976
Smart library			1.0000	0.1189	0.1153	0.1114	0.1380	0.0000
Big data era				1.0000	0.1645	0.0715	0.0492	0.0255
Data mining					1.0000	0.1078	0.0557	0.0000
Information service						1.0000	0.0000	0.1002
Cloud computing							1.0000	0.0345
Digital library								1.0000

**Table 6:** Dissimilarity matrix of the top 30 high-frequency keywords (partial).

	Big data	Library	Smart library	Big data era	Data mining	Information service	Cloud computing	Digital library
Big data	0.0000	1.0000	0.9188	0.9566	0.8821	0.8975	0.8589	0.9028
Library		0.0000	0.9024	0.8607	0.9869	0.9391	1.0000	0.9024
Smart library			0.0000	0.8811	0.8847	0.8886	0.8620	1.0000
Big data era				0.0000	0.8355	0.9285	0.9508	0.9745
Data mining					0.0000	0.8922	0.9443	1.0000
Information service						0.0000	1.0000	0.8998
Cloud computing							0.0000	0.9655
Digital library								0.0000

## Data Availability

The labeled datasets used to support the findings of this study are available from the author upon request.
